# The impact of extended release dopamine agonists on prescribing patterns for therapy of early Parkinson’s disease: an observational study

**DOI:** 10.1186/2047-783X-18-60

**Published:** 2013-12-21

**Authors:** Clelia Pellicano, Dario Benincasa, Alessandra Fanciulli, Pamela Latino, Morena Giovannelli, Francesco E Pontieri

**Affiliations:** 1 Department of Neuroscience, Mental Health and Sensory Organs – (NESMOS), Sapienza University, Via di Grottarossa, 1035-00189, Rome, Italy; 2 Movement Disorder Unit, Sant’Andrea Hospital, Via di Grottarossa, 1035-00189, Rome, Italy; 3 Scientific Institute for Research, Hospitalization and Health Care (IRCSS), Fondazione Santa Lucia, Via Ardeatina, 306-00179, Rome, Italy

**Keywords:** Dopamine agonists, Extended release, Levodopa, Parkinson’s disease, Pramipexole, Ropinirole, Rotigotine

## Abstract

**Background:**

Dopamine agonists (DA) are the first-choice drug for treatment of the early stage of Parkinson’s disease (PD) in subjects younger than 70 years. Recently, a number of third generation DA have been marketed, including transdermal patch of rotigotine and extended release oral formulation of ropinirole and pramipexole.

We investigated the impact of third generation DA on management of the early stage of PD in an outpatient service for Movement Disorders in Italy.

**Methods:**

Two 12-month observation periods were selected (January - December, 2007, and January - December, 2011) as representative for prescription of immediate and extended release formulations of DA respectively. Within each period, PD patients were divided into subgroups according to age (<65 years; 65–75 years; >75 years) or functional requirement (high; moderate; low). For each period, the number of subjects receiving monotherapy with DA, monotherapy with levodopa (LD), or combined DA/LD therapy and the relative doses were calculated. The severity of parkinsonian motor symptoms was calculated by means of the Unified Parkinson’s Disease Rating Scale part III (UPDRS-III) score. The frequency and severity of side-effects leading to discontinuation or reduction of DA drugs at each time point were also calculated.

**Results:**

We found a significant reduction of daily LD dose (both as mono- and combined therapy) between the second and the first observation period. There was also a significant increase of monotherapy with DA and corresponding reduction of monotherapy with LD in patients aged 65–75 years, as well as in PD patients with moderate functional requirements. A significant reduction of frequency of side-effects was measured with extended release DA as compared to immediate release formulations. There were no significant differences of the UPDRS-III scores between the 2 observation periods in any subgroup.

**Conclusions:**

Our results suggest that extended release DA might optimize therapeutic management of the early stages of PD even in patients older than 70 years of age.

## Background

Dopamine agonists (DAs) are the first-choice drugs for treatment of the early stage of Parkinson’s disease (PD) in patients younger than 70 years of age [1]. Several pharmacokinetic and pharmacodynamic properties of DAs [2], including the lack of competition with dietary amino acids upon crossing of intestinal and blood–brain barrier, the relatively long striatal half-life, the lack of metabolism and the direct action at postsynaptic dopamine receptors, contribute to their therapeutic efficacy with reduced risk of motor complications (fluctuations and dyskinesia) compared to levodopa (LD) [3]. Despite these potential advantages, administration of DAs to PD patients is frequently limited by peripheral (cardiovascular and/or gastrointestinal) or central (neuropsychiatric and/or cognitive) side effects [4].

In the past several years, a number of third-generation DAs have been marketed, including a transdermal formulation of rotigotine (RT) and extended-release oral formulations of pramipexole (PP) and ropinirole (RP). These nonergolinic DAs enable continuous stimulation of dopamine receptors that more closely resembles physiological dopaminergic transmission in the basal ganglia [5]. Transdermal RT is efficacious in early stages of PD [6], and extended-release PP and RP show similar therapeutic efficacy as immediate-release formulations [7,8] and reduction of peak-dose side effects [7-9]. Moreover, the once-daily administration regimen improves adherence to the treatment schedule [10]. Taken together, these features suggest that extended-release formulations may increase utilization of DAs in PD patients and thus contribute to further sparing of LD use.

In the present study, we retrospectively investigated the impact of third-generation DAs on prescribing patterns in the early stages of PD by collecting data from patients referred to our Movement Disorder Outpatient Service during two periods of time, before and after marketing of extended-release DAs.

## Methods

We conducted a retrospective study of PD patients recruited sequentially during scheduled visits at the Outpatient Service for Movement Disorders, Mental Health and Sensory Organs Department, Sant’Andrea Hospital, Sapienza University of Rome. In all patients, the PD diagnosis was made according to international guidelines, including sustained response to dopaminergic medications [11]. Two 12-month periods were selected (1 January 2007 through 31 December 2007 and 1 January 2011 through 31 December 2011) as representative for prescription of immediate- and extended-release formulations of DAs, respectively. The protocol was approved by the Ethical Committee of the "Fondazione Santa Lucia IRCCS" and each subject signed an informed consent at enrollment.

The inclusion criteria were (1) Mini Mental State Examination score ≥27; (2) Hoehn and Yahr (H&Y) scale stage ≤2 throughout each observation period; (3) Unified Parkinson’s Disease Rating Scale part III (UPDRS-III) score ≤30; (4) lack of motor and/or nonmotor fluctuations throughout the observation period, investigated by the clinical interview based on the items in the nine-item Wearing-off Questionnaire [12]; and (5) at least two visits during each observation period.

The exclusion criteria were (1) major medical illnesses that may have interfered with antiparkinsonian therapy choice; (2) comorbidity with major psychiatric disorders; (3) history of alcoholism or drug dependence or abuse; (4) neuroradiological (computed tomography or magnetic resonance imaging scan) evidence of significant focal abnormalities; and (5) enrollment in clinical pharmacological trials.

For each participant, the pharmacological therapy used (drugs, formulation and daily doses) at the last visit of each 12-month period was taken as representative of the period itself. Within each 12-month period, eligible patients were divided into three subgroups according to their age (<65 years, between 65 and 75 years and >75 years) and three other subgroups according to their functional requirements (high functional requirement, defined as still at work or involved in regular daily activities; moderate functional requirement, defined as being retired but with regular interests and/or occupations; and low functional requirement, defined as retirement alone). For each subgroup, we calculated the number of patients receiving monotherapy with DAs, monotherapy with LD or combined DA-LD therapy and the relative doses. For DA drugs, the following conversion parameters were applied to calculate LD equivalents: 100 mg of LD = 1 mg of PP = 5 mg of RP = 5 mg RT [7,13]. In the case of combined therapy, the total daily LD equivalent was calculated by adding daily LD (in milligrams) to daily LD equivalents due to DA drugs. Within each 12-month period, the number of patients experiencing side effects that forced modification of drug therapy was also calculated.

Comparisons of continuous variables (sociodemographic features and daily doses of dopamine replacement therapy) were analyzed using a two-tailed, unpaired Student’s *t*-test. As to categorical variables (presence or absence of DAs and presence or absence of significant side effects), the χ^2^ test was applied to analyze differences between the two periods of investigation.

## Results

As shown in Table 1, the two groups did not differ with regard to age, sex, disease stage measured by the H&Y scale and severity of parkinsonian symptoms measured by the UPDRS-III scale. There were no intersubgroup differences in the UPDRS-III scores between the two observation periods (Table 1). As mentioned in the Methods Section, patients did not experience motor fluctuations and/or dyskinesia. There were no patients receiving controlled-release LD and/or amantadine. At each observation period, ten patients were taking rasagiline (1 mg/day). In accordance with the current international guidelines for therapy in the early stages of PD [1], no patients were treated with deep brain stimulation.

**Table 1:** **Demographics and clinical features of the enrolled patients **^**a**^

**Demographics and clinical features**	**Year 2007**	**2011**
*N* (males)	56 (32)	72 (38)
Age, years (mean ± SD)	66 ± 10	69 ± 9
Disease duration, years (mean ± SD)	3.5 ± 1.8	4.6 ± 1.4
Hoehn and Yahr stage (mean ± SD)	1.8 ± 0.4	1.9 ± 0.3
UPDRS-III score (mean ± SD)	20.8 ± 6.1	20.5 ± 6.5
Age <65 years, *n* (%)	20 (35%)	23 (32%)
Age <65 years, UPDRS-III score (mean ± SD)	19.7 ± 3.9	19.3 ± 5.1
Age between 65 and 75 years, N (%)	30 (54%)	31 (43%)
Age between 65 and 75 years, UPDRS-III score (mean ± SD)	20.1 ± 6.7	21.0 ± 5.9
Age >75 years, *n* (%)	6 (11%)	18 (25%)
Age >75 years, UPDRS-III score (mean ± SD)	23.9 ± 5.1	23.5 ± 4.6
High functional requirement, n (%)	18 (32%)	24 (33%)
High functional requirement, UPDRS-III score (mean ± SD)	20.2 ± 6.8	20.9 ± 5.9
Moderate functional requirement, n (%)	20 (36%)	19 (26%)
Moderate functional requirement, UPDRS-III score (mean ± SD)	22.1 ± 5.2	21.9 ± 4.8
Low functional requirements, n (%)	18 (32%)	29 (40%)
Low functional requirement, UPDRS-III score (mean ± SD)	24.1 ± 5.2	24.4 ± 4.9
Daily LD, monotherapy, mg (mean ± SD)	328 ± 67	267 ± 62^b^
Daily DA equivalents, monotherapy, mg (mean ± SD)	237 ± 74	277 ± 62
Daily total LD equivalents, combined therapy, mg (mean ± SD)	483 ± 133	440 ± 111
Daily DA equivalents, combined therapy, mg (mean ± SD)	161 ± 80	177 ± 78
Daily LD, combined therapy, mg (mean ± SD)	330 ± 72	263 ± 61^b^
Side effects forcing reduction/withdrawal of DA therapy, *n* (%)	7/37 (18.9%)	7/57 (12.3%)^c^

^a^DA, dopamine agonist; LD, levodopa; UPDRS-III, Unified Parkinson’s Disease Rating Scale part III. ^b^*P* < 0.01 different from 2007 by two-tailed, unpaired Student’s *t*-test. ^c^*P* < 0.01 different from 2007 by χ^2^ test. See Methods Section for details.

In the whole patient population, there was a significant reduction in the daily LD dose between the second and the first periods of observation (267 ± 62 mg vs. 328 ± 67 mg for patients on monotherapy with LD; 263 ± 61 mg vs. 330 ± 72 mg for patients on combined therapy with LD and DA) (Table 1). Moreover, in 2007, the DA dose was increased in seven patients (19%) and reduced in six patients (15%). Conversely, in 2011, DA dose was increased in ten patients (18%) and was decreased in six patients (10%).

Analysis of age-related subgroups indicated the significant increase of monotherapy with DAs (45% vs. 14%) and reduction of monotherapy with LD (6% vs. 37%) in patients aged between 65 and 75 years between the second and the first observation period (Table 2). In this subgroup of patients, there was also a significant increase of dosage of DAs, measured as daily LD equivalents (314 ± 53 mg vs. 250 ± 57 mg) (Table 2).

**Table 2:** **Distribution of dopamine replacement therapy according to patient age**^**a**^

**Patient age**	**Therapy**	**2007**	**Year 2011**
Age <65 years	DA monotherapy, *n* (%)	10 (50%)	14 (61%)
	Daily LD equivalents, mg (mean ± SD)	245 ± 52	281 ± 48
	LD monotherapy, *n* (%)	3 (15%)	2 (9%)
	Daily mg (mean ± SD)	274 ± 29	275 ± 15
	DA + LD combined therapy, *n* (%)	7 (35%)	7 (30%)
	Total daily LD equivalents, mg (mean ± SD)	385 ± 62	388 ± 70
Age between 65 and 75 years	DA monotherapy, *n* (%)	4 (14%)	14 (45%)^b^
	Daily LD equivalents, mg (mean ± SD)	250 ± 57	314 ± 53^b^
	LD monotherapy, *n* (%)	11 (37%)	2 (6%)^b^
	Daily dose, mg (mean ± SD)	325 ± 50	350 ± 25
	DA + LD combined therapy, *n* (%)	14 (47%)	15 (49%)
	Total daily LD equivalents, mg (mean ± SD)	425 ± 40	415 ± 54
Age >75 years	DA monotherapy, *n* (%)	0 (0%)	1 (6%)
	Daily LD equivalents, mg (mean ± SD)		250 ± 0
	LD monotherapy, *n* (%)	4 (67%)	11 (61%)
	Daily dose, mg (mean ± SD)	465 ± 28	450 ± 20
	DA + LD combined therapy, *n* (%)	2 (33%)	6 (33%)
	Total daily LD equivalents, mg (mean ± SD)	525 ± 25	530 ± 22

^a^DA, dopamine agonist; LD, levodopa. ^b^*P* < 0.01 compared with 2007 by χ^2^ statistic or unpaired Student’s *t*-test statistic. See Methods Section for details.

We found a significant increase in monotherapy with DAs (53% vs. 25%) and a significant reduction in monotherapy with LD (10% vs. 35%) between the second and first observation periods among patients with moderate functional requirements (Table 3). In this subgroup, the daily dose of DAs, expressed as LD equivalents, were significantly higher in 2011 (325 ± 33 mg) than in 2007 (250 ± 25 mg) (Table 3).

**Table 3:** **Distribution of dopamine replacement therapy according to patients’ functional requirements**^**a**^

**Function level**	**Therapy**	**2007**	**2011**
High	DA monotherapy, *n* (%)	6 (33%)	14 (59%)^b^
	Daily LD equivalents, mg (mean ± SD)	350 ± 57	335 ± 57
	LD monotherapy, *n* (%)	3 (17%)	2 (8%)
	Daily dose, mg (mean ± SD)	315 ± 33	325 ± 15
	DA + LD combined therapy, *n* (%)	9 (50%)	8 (33%)
	Total daily LD equivalents, mg (mean ± SD)	400 ± 52	415 ± 35
Moderate	DA monotherapy, *n* (%)	5 (25%)	10 (53%)^b^
	Daily LD equivalents, mg (mean ± SD)	250 ± 25	325 ± 33^b^
	LD monotherapy, *n* (%)	7 (35%)	2 (10%)^b^
	Daily dose, mg (mean ± SD)	280 ± 25	275 ± 12
	DA + LD combined therapy, *n* (%)	8 (40%)	7 (37%)
	Total daily LD equivalents, mg (mean ± SD)	324 ± 34	330 ± 35
Low	DA monotherapy, *n* (%)	3 (17%)	4 (14%)
	Daily LD equivalents, mg (mean ± SD)	255 ± 15	261 ± 27
	LD monotherapy, *n* (%)	9 (50%)	12 (41%)
	Daily dose, mg (mean ± SD)	250 ± 25	230 ± 32
	DA + LD combined therapy, *n* (%)	6 (33%)	13 (45%)
	Daily LD equivalents, mg (mean ± SD)	289 ± 21	277 ± 27

^a^DA, dopamine agonist; LD, levodopa. ^b^*P* < 0.01 compared with 2007 by χ^2^ test or unpaired Student’s *t*-test. See Methods Section for details.

In 2007, moderate to severe side effects were recorded in 7 (18.9%) of 37 patients treated with DAs (monotherapy or combined therapy) (Table 1). These side effects included daytime sleepiness (*n* = 3), visual hallucinations (*n* = 2), impulse control disorder (ICD) (*n* = 1) and cognitive impairment (*n* = 1). In two of these cases, the severity of side effects forced withdrawal of DA therapy. In the remaining five cases, adverse side effect symptoms were controlled by reducing the DA dose. Side effects were detected in patients younger than age 65 (*n* = 2) and those between 65 and 75 years of age (*n* = 5). Conversely, in 2011, 7 (12.3%) of 57 patients receiving therapy with DAs experienced moderate to severe side effects (Table 1), including daytime sleepiness (*n* = 3), ICD (*n* = 3) and visual hallucinations (*n* = 1). In only one case, the severity of the side effect prompted us to suspend DAs. In the remaining cases, adverse symptoms were controlled by reducing doses of DAs. Side effects were reported in one patient aged younger than 65 years of age, in five between 65 and 75 years of age and in one patient older than age 75 years. There was a 35% reduction in the occurrence of side effects in 2011 compared to 2007 (*P* < 0.01) (Table 1).

## Discussion

We carried out this retrospective, observational study of a homogeneous cohort of patients (drawn from patients referred to our Outpatient Service for Movement Disorders) to evaluate the impact of introduction of extended release DAs on prescription patterns in the early, uncomplicated, stages of PD. We are aware of several limitations of this study, including the small sample size and the lack of data on therapeutic adherence and treatment satisfaction among our patients. However, the very similar demographic and clinical features of the two populations enrolled allowed us to identify significant differences that might have an impact on therapeutic management of patients in the early stages of PD.

The results show that introduction of extended-release DAs was accompanied by significant reductions in daily LD doses (Table 1) and a decrease in side effects that would have required a reduced dose or withdrawal of DA drugs (Table 1). The prevalence of moderate to severe side effects associated with extended-release DAs in our patients is similar to that reported recently by other authors [14]. Cumulatively, these findings suggest that marketing of extended-release DAs contributes significantly to modifying therapeutic strategies for early PD patients referred to our institution. Indirectly, these changes allowed stricter adherence to the current therapeutic guidelines for uncomplicated PD [1] and are in accord with a recent report from France [15].

Our results show increased prescription of DAs in 2011 compared to 2007 in most subgroups (Tables 2 and 3). In particular, it is of interest that a significant increase in monotherapy with DAs, coupled with significantly reduced monotherapy with LD, was found in patients between 65 and 75 years of age (Table 2). Within this age group, DAs were prescribed (as monotherapy or in combination with LD) in more than 90% of cases in 2011 compared to 62% of cases in 2007. We think the increased use of DAs and the reduction in LD therapy occurred in this group of patients, and not in younger patients, because younger patients were already receiving higher dosages of DAs. These findings suggest that extended-release formulations of DAs may contribute significantly to delaying LD prescriptions and/or to reducing daily LD dosages for patients older than 70 years of age as well. If confirmed by further studies with larger cohorts, these results may suggest consideration of monotherapy with DAs or combined DA-LD therapy as the preferred approach to treatment of patients with uncomplicated PD younger than 75 years of age.

A further relevant observation of the present study is related to the analysis of subgroups identified according to functional requirements (Table 3). In subjects with moderate functional requirements, significant increases of monotherapy with DAs and significant reductions of monotherapy with LD were found in 2011 compared to 2007. Similar trends were observed in patients with high functional requirements, although among the latter cohort, significance was reached for monotherapy with only DAs. In particular, in this latter subgroup, the most frequently prescribed therapy was combined LD and DA in 2007 (50% of cases) and monotherapy with DAs in 2011 (59% of cases).

Moreover, it is interesting to note that there was a discrete relationship between the results in the age-related and functional requirement–related subgroups. We think this latter finding probably reflects more requests for improved function among younger patients. In this respect, it is notable that the significantly increased prescription of monotherapy with DAs in patients carrying out daily professional and/or personal activities may be related to the higher daily doses of extended-release DAs in 2011 compared to immediate-release formulations in 2007 (Table 3). In turn, this may reflect higher tolerability (that is, reduced peak-dose side effects) of extended-release formulations than immediate-release DAs [8-10].

## Conclusions

The results of the present study suggest that extended-release DAs can be substituted for immediate-release DAs with less side effects and can contribute to sparing use of LD. These findings are in line with the results of previous randomized trials of extended-release DAs [7-9] in patients with uncomplicated PD. Moreover, the introduction of extended-release DAs may contribute to widening the prescription of these drugs as monotherapy or in combination with LD for patients older than 70 years of age and still engaged in intense or regular daily activities. Further studies using more detailed methodologies with larger sample sizes are needed to confirm these preliminary findings, as well as to investigate the post-marketing role of extended extended-release DAs in patients with more advanced stages of PD.

## Abbreviations

DA: Dopamine agonist; H&Y: Hoehn and Yahr; LD: Levodopa; PD: Parkinson’s disease; PP: Pramipexole; RP: Ropinirole; RT: Rotigotine; UPDRS-III: Unified Parkinson’s Disease Rating Scale part III.

## Competing interests

The authors declare that they have no conflicts of interest.

## Authors’ contributions

CP conceived the study, participated in its design, collected data and wrote the first draft of the manuscript. DB, AF and PL participated in the design of the study, collected data and critically reviewed the first draft of the manuscript. MG participated in the design of the study, performed the statistical analysis and critically reviewed the first draft of the manuscript. FEP conceived the study, participated in the study design and coordination and critically reviewed the first draft of the manuscript. All authors read and approved the final manuscript.
